# Knee Surgery during the COVID-19 Lockdown—Experiences of a Level-One Trauma Center in Germany

**DOI:** 10.1155/2021/8875643

**Published:** 2021-05-25

**Authors:** Matthias Koch, Daniel Popp, Viola Freigang, Borys Frankewycz, Katja Hierl, Peter Angele, Volker Alt, Michael Worlicek

**Affiliations:** ^1^Department of Trauma Surgery, University Medical Centre Regensburg, Regensburg, Germany; ^2^Sporthopaedicum, Regensburg, Germany

## Abstract

**Background:**

Almost every sector in the health care is affected by the COVID-19 pandemic. Many studies already investigated the effect on different aspects in orthopedic and trauma care. However, the current literature lacks data regarding the consequence on daily surgical business. Thus, the aim of the present study was to analyze the development of knee-related pathologies and surgical procedures in a German university level-one trauma center during the lockdown phase and early lockdown phase to investigate the impact of the COVID-19 lockdown on orthopedic and trauma knee surgery. *Material and Methods*. The amount of knee joint surgeries performed during the high-peak COVID-19 crisis in the period of January to May 2020 was evaluated retrospectively and compared to the corresponding time periods of the previous years (2017-2019).

**Results:**

The COVID-19 lockdown led to a significant decrease in the number of knee injuries in March and April 2020 by 83.3%. Surgical procedures were reduced by 84.8% during the same period. In May 2020, the number of knee joint procedures returned to an almost prepandemic level. The distribution of urgent and elective knee surgery changed to predominantly acute trauma care at the beginning of the COVID-19 lockdown and persisted through to May 2020.

**Conclusion:**

The COVID-19 pandemic had a high impact on emergency and elective knee surgery in a level-one trauma center in Germany during the lockdown phase. It also showed that a level-one trauma center in the German healthcare system is able to handle urgent trauma and orthopedic operations during a worldwide medical crisis and to return to a prepandemic level within a short phase.

## 1. Introduction

The coronavirus disease 2019 (COVID-19) pandemic caused severe changes to health systems and daily routines worldwide [1–3]. Based on the experiences of China and later on in Italy, radical and wide measures were taken to minimize the risks of COVID-19-related hazards. Many European governments announced a total lockdown to reduce the dissemination and incidence of the COVID-19 disease. The first case in Germany was documented on January 27^th^, 2020 [4]. Due to the rapid increase of the incidence and limited therapy options, a total lockdown, including wide restrictions on outdoor activities and personal contacts, as well as shutdown of restaurants and stores, was decreed on March 13^th^, 2020. In Bavaria, the complete lockdown for the public and private sector was announced on March 20^th^, 2020. Private meetings outside the family were restricted, and leaving the house was only allowed for necessary actions like food shopping. Visiting of hospitals and nursing homes was prohibited. In addition to the economic sector, the health care system was also significantly hit by this historical cutback. Due to the expected medical capacity requirements for the treatment of COVID-19 patients, all medical services were reduced to essential health care [5, 6]. The decreed public cutback decisions were relaxed step by step beginning on April 20^th^ with an opening permission for stores with more than 800 square meters of size until lockdown restrictions were abolished on May 6^th^, 2020, with an achievement of an almost normal daily routine. Medical services that returned to daily routine adapted to the local COVID-19 situation in a time-displaced manner [7].

During the period of the COVID-19 lockdown for trauma and orthopedic surgeons, there was clear advice to reduce the outpatient department workflow and elective surgeries [4, 8, 9]. Nevertheless, trauma emergency surgery was necessary due to its essential role in patient care. Regarding the current literature, there are many studies available investigating the effect on different aspects in orthopedic and trauma care, such as triage of orthopedic and trauma diseases, management of orthopedic and trauma surgery during the pandemic, as well as the return after lockdown phase, postoperative surveillance of orthopedic and trauma patients, and educational aspects regarding residents during the pandemic [10–14]. Also, the impact of the COVID-19 pandemic was already investigated on survey-based studies [4, 8, 9]. However, the literature lacks sufficient data regarding the impact of the COVID-19 pandemic on orthopedic and trauma surgery as measured by real surgery data.

Knee surgery, as a definable subcategory of orthopedic and trauma surgery, is characterized by a broad overlapping of orthopedic and trauma indications for elective and acute surgery. Thus, this study analyzes the development of knee-related pathologies and surgical procedures in a German university level-one trauma center during the lockdown phase and early lockdown phase to investigate the impact of the COVID-19 lockdown on orthopedic and trauma surgical business.

## 2. Material and Methods

### 2.1. Study Design and Patient Selection

In this retrospective epidemiological study, all surgical procedures regarding knee joint pathologies in a German university level-one trauma center within the period of January to May 2020 were analyzed per month in accordance to the criteria listed in Table 1. The same months of 2017, 2018, and 2019 served as a control (averaged per month). The design and methods of this study were approved by the University's Ethical Committee (Ethical Grant Number: 20-1872-104). All knee surgeries performed during the above mentioned period were included in the present study.

### 2.2. Management during COVID-19 Pandemic

The management of the COVID-19 pandemic was headed by a hospital task force including representatives of all medical departments, nursing care, and administration. By daily evaluation of the pandemic situation, a flexible adaption to the current situation was ensured.

In the early March, when COVID-19 pandemic impended to reach Germany, an enlightenment of all employees was performed, and additional trainings were accomplished to improve and refresh intensive care knowledge of the medical staff (nurses and physicians) and to also flexibly deploy surgeons and other specialists to support the treatment of COVID-19 patients on special COVID-19 wards and intensive care units.

In mid-March, access to the university medical center was limited to patients requiring acute treatment. All patient admissions took place via the emergency room, where COVID-19 screening was performed. Additionally, consequent wearing of cloth face masks was decreed. In front of the emergency room, a triage of patients suspicious for COVID-19 and no-COVID-19 suspicious was performed, and a further separation followed in the emergency room and eventually in the ward. All patients were tested for a COVID-19 infection. COVID-19 suspicious patients were initially treated on special COVID-19 wards, until negative COVID-19 test results were received. Remaining patients could be treated on the normal ward.

Regarding surgical therapy, the operating room capacities were reduced by the task force to emergency surgery only to save medical resources. Patients with indication for acute surgery, including fractures, knee dislocation, or dislocated bucket-handle tear of the meniscus, were triaged to immediate and urgent emergency indication for surgical therapy. In case of immediate indication for surgical intervention, such as applying external fixator, fasciotomy, or septic arthritis, COVID-19 testing was not performed, and surgery was conducted according to the official recommendations for treating COVID-19 patients 24/7. In case of urgent indication for surgery, such as osteosynthesis or knee stabilization after dislocation, COVID-19 test results were waited for. These results were generally received by no later than 24 hours, and surgery was planned for daily emergency business in agreement with the other surgical departments. Emergency surgery capacities were increased in line with the increasing demands after official lockdown reduction at the end of April before elective surgery restarted in a time-displaced from mid of June. Common with the emergency patients, all elective surgery patients are now screened concerning a COVID-19 infection before surgery.

### 2.3. Statistical Analysis

Descriptive analysis was performed using SPSS® (Version 25, IBM, Armonk, NY, USA). Mean values and standard deviations were calculated for each consecutive month of the control year (January, February, March, April, and May) and compared to absolute values of the COVID-19 pandemic period of January to May 2020.

## 3. Results

The COVID-19 lockdown in April 2020 was associated with a clear decrease of almost three quarters in the number of patients treated for knee injuries in comparison to the respective periods of the previous three years. Furthermore, the ratio of elective and acute surgeries changed to predominantly acute trauma and orthopedic care of knee joint pathologies during this period. Overall, one treated patient was known to be COVID-19 positive during the knee injury therapy (septic arthritis of both knee joints; Table 2 gives an overview of the demographic data).

Even if the number of knee injuries was clearly reduced during the COVID-19 lockdown, no relevant changes in the injury pattern could be detected due to the small sample size (see Table 3). The evaluation showed overall a high monthly variance of total number of knee pathologies, which was topped in March and April 2020 with an overall reduction of up to 83.3%.

In spite of a high monthly variance of knee surgeries, a clear decrease of surgical procedures could be detected in March (almost one-third) and in April 2020 (almost 85%). During the lockdown period in March and April, knee surgery was reduced to emergency surgery. These operations included joint revision in case of septic arthritis and osteosynthesis in case of femur/tibia/patella fracture. Also, soft tissue procedures were performed like patellar tendon refixation after traumatic rupture, meniscus refixation combined with anterior cruciate ligament reconstruction in case of a traumatic dislocated bucket-handle tear, and anterior cruciate ligament rupture associated with severe hemarthrosis and subjective instability. In May 2020, the number of procedures returned to an almost prepandemic level (see Table 4).

## 4. Discussion

The main finding of this study was that the COVID-19 pandemic-caused lockdown, which was declared in Germany and in most parts of Europe during spring 2020, led to a decrease of surgical knee joint procedures in March and especially in April 2020. While in March 2020 the amount of inpatient knee joint surgeries was reduced almost one-third in comparison to the mean values of the corresponding months of the three previous years, in April 2020, the number of knee surgeries decreased by 85%.

Although a slight reduction in knee operations was also found in January and February compared to the respective mean values of previous years, regarding the respective standard deviations, this has to be considered a normal monthly variance of surgically treated knee diseases. In contrast to that, the clear reduction in March and especially April 2020 emphasizes the massive impact of the COVID-19 pandemic and associated lockdown on the knee surgery. The evaluated data also shows that a clear majority of procedures performed during this period had acute urgency. Thus, this study supports preliminary survey-based reports of a massive cutback in orthopedic health care services due to COIVD-19 pandemic [4, 8]. However, it also reflects the essential relevance of trauma and orthopedic care for the health care system by keeping trauma and orthopedic surgery in business, even in a reduced manner. The COVID-19 pandemic with its complete lockdown has been unique in modern medicine [15]. Thus, there are no validated historical data and no actual data yet available to predict the real impact of such a pandemic on the health care system, especially on elective inpatient surgery and emergency inpatient surgery. Regarding the current literature, there is just one recent study available investigating the influence of the pandemic on elective orthopedic surgery, like arthroplasty and spine fusion surgery in the United States of America based on a stochastic simulation [15]. This study predicted that in an optimistic estimate, it will take over six months for the US healthcare system to return to 90% of its prepandemic level of elective inpatient orthopedic surgery. The evaluated data in this study show an accelerated return to prepandemic business in trauma and orthopedic surgery. Reducing of the lockdown measures at the end of April and beginning of May 2020 was associated with a clear increase of knee-related pathologies as well as knee joint procedures to a number similar to that of the previous years. However, the distribution of acute and elective surgery was still predominantly in favor of acute knee trauma therapy. Contemporary literature lacks data regarding the distribution of knee procedures, especially for elective or acute trauma and orthopedic surgeries in relation to the season. In consequence, it is unknown if there is a COVID-19-independent increase of acute trauma and orthopedic surgery in the early summer time. The increase of acute treated knee trauma cases might have rather been caused by an increased accident rate directly after reducing the COVID-19-related restrictions, which will probably be detected in future epidemiological studies. This would support the prediction by Jain et al. of a decelerated return of elective orthopedic surgery after COVID-19 lockdown caused by an increasing need for acute orthopedic and trauma surgery [15].

Regarding other surgical specialties, massive restrictions by the COVID-19 pandemic are described. For example, Lechner et al. analyzing the impact of COVID-19 pandemic on a visceral surgical department in Austria detected an increase of emergency operations associated with a clear decrease of oncological operations [16]. Also, Stoss et al. evaluating the impact of the pandemic situation on nonuniversity surgical departments proved the special character of this unique occasion [17]. The reduced number of surgeries was caused not only by the decreed restrictions but also by uncertainties of afraid patients, who canceled their surgery appointments. Overall, these reservations regarding inpatient procedures are basically reasonable regarding the COVID-19 pandemic situation.

At the time of this study, the number of COVID-19 infections per capita was much higher in the United States compared to Germany. At that time, the latest statistics of the Johns Hopkins University showed over 2,000,000 confirmed infections in the United States and approximately 186,000 confirmed infections in Germany [18, 19]. Although the consistent policies in Germany most likely helped to contain the spreading of the virus more successfully, there were some hot spots with an average higher number of COVID-19 infections like East Bavaria. By consequence, the investigated level-one trauma center, located within one of these areas, had to treat a high number of COVID-19 positive patients. During the peak of the outbreak, there were 43 patients treated simultaneously, of which 36 required ventilation and 15 required extracorporeal membrane oxygenation (ECMO). Even though a high proportion of the hospital's medical capacity was in use, a certain capability was assigned to surgeries. However, even if the presented numbers of surgical knee joint procedures suggest an accelerated return to prepandemic status in a level-one trauma center, the distribution of acute to elective surgery supports the study of Jain et al., predicting a slow return to prepandemic elective orthopedic surgery, which require established algorithms that guarantee safety of the patients and medical staff [15].

However, the development of such algorithms across all disciplines is influenced by the uncertainties and problems regarding the safety of surgical techniques or also the availability and use of personal protective equipment (PPE). For example Saverio et al. reported that there might be a higher spread of the virus using laparoscopy, because of aerosolization due to pneumoperitoneum and to heat-generating cautery devices [20]. In consequence, the authors recommend to use laparotomy, if awaiting the results of COVID-19 testing would delay an urgent operation. Also, regarding arthroscopy, which is mainly used in elective surgery and where conversion to open surgery is usually not a relevant option, the risk of surgery is not clear, what also may decelerate the return to the “normal status”.

While in case of elective surgery a risk-reduction for medical staff can be expected due to testing of the patients, in emergency procedures, a fast risk assessment is required. In this context, the different symptoms of a possible COVID-19 infection have to be considered. Thus, based on the basic pathomechanisms of a COVID-19 infection and possible absence of respiratory symptoms [21], Lima et al. recommended an additional chest CT for patients with acute abdomen [22]. In the case of knee injuries, however, the additional radiation is not that easily justified.

Nevertheless, even if the risk of COVID-19 infection in the patients can be reduced by tests and checklists, a residual risk remains for the patient and the medical staff. Until all medical staff has been vaccinated, PPE is and will be a permanent accompanist in emergency surgery as well as elective surgery. This is also an important factor for the development of algorithms that needs to be taken into account. The COVID-19 pandemic claimed the use of new and unaccustomed PPE during surgery. However, according to a survey by Benitez et al. assessing team organization, PPE-related aspects, operation room preparations, anesthesiologic considerations, and surgical management for emergency surgery during the pandemic showed problems regarding the availability and use of PPE [23]. About half of the respondents indicated to have a scarcity or even absence of protective equipment, and also, almost half of the respondents had not received training in the use of PPE while performing emergency surgical procedures before the pandemic. Accordingly, also about half of the respondents did not feel adequately protected by the PPE. Furthermore, a recent survey among surgeons from 26 countries showed that surgeons felt that their surgical performance was hampered by using PPE. Visual impairment and problems with communication were also reported [24], which might have an impact on the surgical outcome.

Overall, these are challenging factors, which have to be considered and solved by future algorithms before a complete return to the prepandemic level can be reached.

Regarding the current literature, the first recommendations by the World Health Organization (WHO) and similar organizations have been adopted globally by surgery departments, including the restructuring of surgical schedules, staff preparation, the department outbreak response protocols, and recommendations for surgical techniques and risk management [25]. This shows that first lessons have been learned from this crisis, but further steps have to be followed. Certainly, this study has some limitations. Firstly, only one German level-one trauma center has been evaluated. Therefore, the applicability of those findings is limited, and the impact on the whole trauma and orthopedic surgery sector of Germany or other countries needs to be investigated in broader studies. Secondly, the study focuses on analyzing knee joint-related surgeries only. Even though this data can be assumed a valid representation of the distribution of acute and elective surgery within a trauma and orthopedic center, the impact on the overall trauma and orthopedic care needs to be done with caution.

## 5. Conclusion

This study showed that the COVID-19 pandemic had a high impact on emergency and elective knee joint surgery in a level-one trauma center in Germany during the lockdown phase. Knee-related pathologies as well as knee surgery significantly decreased in accordance to the public lockdown instructions. However, the data also showed that orthopedic and trauma surgery, and especially knee surgery, is relevant for the health care system so that even during the crisis, knee surgery was performed. After relaxation of the lockdown, knee-related pathologies and knee surgery resumed to an almost prepandemic level, but with predominantly acute orthopedic and trauma surgery, probably due to a reactive increase of accidents. Although the German health care system was able to handle this historical crisis so far, guidelines for managing a pandemic during and after such a lockdown phase are necessary.

## Figures and Tables

**Table 1:** General data.

General data	(i) Number of included patients (ii) Sex (male/female) (iii) Age (years) (iv) Insurance (occupational/normal) (v) Urgency (acute/elective) (vi) Known COVID-19 infection
Type of pathology	(i) Fracture (including proximal tibia/distal femur/patella) (ii) Soft tissue (including ligament, meniscus, tendon, and muscle injuries) (iii) Cartilage injuries (iv) Osteoarthritis (v) Malalignment (vi) Septic (vii) Knee luxation (viii) Tumor
Surgical procedure	(i) Osteosynthesis (ii) Arthroplasty (iii) Reconstructive surgery (including ligament, meniscus, tendon, and muscle therapy + realignment) (iv) Septic surgery (v) Tumor surgery

**Table 2:** General data (Jan: January; Feb: February).

General data	Jan 2017-2019 Mean (SD)	Jan 2020 *n*	Feb 2017-2019 Mean (SD)	Feb 2020 *n*	March 2017-2019 Mean (SD)	March 2020 *n*	April 2017-2019 Mean (SD)	April 2020 *n*	May 2017-2019 Mean (SD)	May 2020 *n*
Number of patients	13.7 (2.9)	11	20.3 (3.2)	21	17.0 (7.2)	12	17.3 (5.7)	4	15.7 (7.2)	15
Sex										
Male	9.7 (3.1)	7	15.3 (1.5)	11	12.7 (7.4)	6	14.3 (5.7)	2	11.0 (1.7)	8
Female	4.0 (1.0)	4	5.0 (2.0)	10	4.3 (0.6)	6	3.0 (0.0)	2	4.7 (5.5)	7
Age	41.2 (7.1)	48.4 (18.2)	45.2 (3.5)	46.7 (21.3)	46.6 (0.8)	47.0 (17.7)	41.4 (1.9)	45.6 (5.2)	45.1 (4.2)	43.4 (23.4)
Insurance situation										
Occupational	5.7 (0.6)	3	9.7 (3.1)	5	4.7 (3.2)	3	4.7 (2.3)	1	2.7 (1.5)	7
Normal	7.7 (3.8)	8	10.7 (5.1)	16	12.3 (4.9)	9	12.7 (3.5)	3	13.0 (7.2)	8
Urgency										
Acute	3.3 (2.3)	3	7.7 (1.2)	7	6.7 (4.0)	6	7.0 (3.5)	3	5.7 (3.2)	8
Elective	10.3 (0.6)	8	12.7 (2.1)	14	10.3 (4.7)	6	10.3 (5.9)	1	10.0 (6.0)	7
Known COVID-19 positive patients	0	0	0	0	0	1	0	0	0	0

**Table 3:** Pathologies (Jan: January; Feb: February).

	Jan 2017-19 Mean (SD)	Jan 2020 *n*	Feb 2017-2019 Mean (SD)	Feb 2020 *n*	March 2017-2019 Mean (SD)	March 2020 *n*	April 2017-2019 Mean (SD)	April 2020 *n*	May 2017-2019 Mean (SD)	May 2020 *n*
Fracture	3.3 (2.5)	4	6.7 (4.2)	7	6.7 (2.1)	3	5.3 (2.5)	2	3.0 (2.0)	5
Soft tissue	8.7 (2.9)	7	9.3 (2.5)	4	7.3 (6.1)	4	9.3 (5.5)	2	10.3 (11.0)	9
Cartilage	2.0 (1.0)	1	3.7 (2.5)	5	1.0 (1.0)	0	2.0 (1.0)	0	1.0 (1.0)	1
Osteoarthritis	0.3 (0.6)	0	2.0 (2.0)	3	0.3 (0.6)	2	1.3 (0.6)	0	1.3 (1.2)	0
Malalignment	0.7 (0.6)	0	0.0	0	1.0 (1.0)	0	0.7 (0.6)	0	0.3 (0.6)	0
Septic	0.0	0	1.3 (1.5)	2	2.7 (0.6)	4	3.3 (2.3)	0	2.3 (1.2)	2
Knee luxation	1.3 (1.5)	1	2.3 (2.5)	0	0.3 (0.6)	0	1.0 (1.0)	0	1.3 (2.3)	0
Tumor	0.0	0	0.3 (0.6)	0	0.3 (0.6)	0	1.0 (1.0)	0	0.0	0
Total	16.3 (5.9)	13	25.7 (3.5)	21	19.7 (10.0)	13	24.0 (11.5)	4	19.7 (12.4)	17
Delta (%)	-20.2		-18.3		-34.0		-83.3		-13.7	

Delta is defined as the percentage difference between the respective total values of the period 2017-2019 versus 2020 (delta = ([value 2020] − [value 2017 − 2019])/100).

**Table 4:** Surgical procedures (Jan: January; Feb: February).

	Jan 2017-2019 Mean (SD)	Jan 2020 *n*	Feb 2017-2019 Mean (SD)	Feb 2020 *n*	March 2017-2019 Mean (SD)	March 2020 *n*	April 2017-2019 Mean (SD)	April 2020 *n*	May 2017-2019 Mean (SD)	May 2020 *n*
Osteosynthesis	3.3 (2.5)	4	7.7 (4.2)	8	8.0 (3.5)	3.0	6.3 (3.2)	2.0	3.7 (1.5)	4.0
Arthroplasty	0.3 (0.6)	0	2.0 (1.7)	4	1.3 (1.5)	3.0	1.7 (0.6)	0.0	0.7 (1.2)	2.0
Reconstructive surgery	15.3 (5.9)	12	18.7 (1.5)	10	10.7 (7.1)	4.0	13.7 (8.4)	2.0	16.0 (8.9)	9.0
Septic surgery	0.0	0	1.0 (1.7)	2	1.7 (1.2)	4.0	3.7 (2.1)	0.0	1.7 (1.2)	4.0
Tumor surgery	0.0	0	0.0	0	0.3 (0.6)	0.0	1.0 (1.0)	0.0	0.0	0.0
Total	19.0 (7.9)	16	29.3 (2.9)	24	22.0 (9.0)	14.0	26.3 (13.6)	4.0	22.0 (10.6)	19.0
Delta (%)	-15.8		-18.2		-36.4		-84.8		-13.6	

Delta is defined as the percentage difference between the respective total values of the period 2017-2019 versus 2020 (delta = ([value 2020] − [value 2017 − 2019])/100).

## Data Availability

Data are available on reasonable request.
